The article "The Effect of PACS in Breast Tumor Diagnosis Based on Numerical Analysis" was published in 2022. Journal: Comput Math Methods Med.

# The Effect of PACS in Breast Tumor Diagnosis Based on Numerical Analysis

**DOI:** 10.1155/2022/7259951

**Published:** 2022-07-13

**Authors:** Guijun Guo, Yi Chen

**Affiliations:** Chongqing Red Cross Hospital (People's Hospital of Jiangbei District) Department of Radiology, Chongqing 400020, China

## Abstract

The incidence and mortality rates are increasing year by year, and the incidence of the disease is gradually becoming younger. The purpose of this study was to investigate the clinical diagnostic value of PACS in breast tumor patients. *Methods*. 20 patients with breast tumor diagnosed by PACS were selected for the study, and the diagnosis was confirmed by pathological puncture or surgery. *Results*. The detection rates of breast tumor by MRI and CT were 94.44% and 96.67%, the sensitivities were 18.82% breast tumor and 96.67%, and the specificities were 53.84% and 54.54%, with no statistically significant difference (*P* > 0.05). There was no statistically significant difference in the detection rate of invasive lobular carcinoma (LDC) and PACS (*P* > 0.05). *Conclusion*. PACS has a greater detection rate for breast tumor and offers some diagnostic usefulness in diagnosing malignant breast tumor. The detection rate of breast tumors can be increased by selecting the most appropriate diagnostic tool for the patient's current circumstances.

## 1. Introduction

The incidence and mortality rates are increasing year by year, and the incidence of the disease is gradually becoming younger [1–3]. In recent years, it has been found that the clinical outcome and prognosis of breast tumor are closely related to different molecular subtypes [4]. In clinical practice, the early identification of molecular subtypes [5].

Breast cancer is a malignant tumor that is genetically heterogeneous. There are some disparities in prognosis due to the varied biological behaviours of different molecular subtypes of breast tumor, which has been a hot issue of research both at home and abroad in recent years [6]. Many studies [7] have shown that the clinicopathological characteristics and prognosis of different molecular subtypes of breast tumor are significantly different. Molecular biology studies have confirmed the role of ER, PR, and HER-2 in the development of breast tumors, making them one of the most important reference indicators for assessing the biological behaviour of cancer cells and developing treatment plans [8]. The molecular pathology of luminal B breast tumor is characterized by ER-positive or/and PR-positive and HER-2 positive or negative but Ki − 67 > 14% [9], and endocrine therapy is effective, while molecularly targeted therapy is feasible due to partial positive HER-2 expression. HER-2 overexpression type is effective for molecular targeted therapy but is prone to metastasis, high recurrence rate, and poor prognosis [10].

The article "The Effect of PACS in Breast Tumor Diagnosis Based on Numerical Analysis" was published in 2022. Journal: Comput Math Methods Med.

The triple negative type is resistant to both endocrine and molecular targeted therapy but is very aggressive and prone to metastasis and has the worst prognosis of all molecular subtypes. Early identification of diverse genetic subtypes of breast carcinoma is therefore critical in clinical practice for early and specific clinical treatment and prognosis [11, 12]. Results from prospective screening trials in European populations have shown that DBT as a stand-alone diagnosis or as an adjunct to digital mammography (DM) increases cancer detection rates by approximately 30% compared to DM alone [13]. The aim of this paper is to analyze the value of combining DM and DBT in the diagnosis of molecular subtypes of breast tumor and to provide a basis for more targeted clinical treatment planning [14].

The paper's organization paragraph is as follows: the related work is presented in Section 2.  Section 3 analyzes the materials and methods of the proposed work.  Section 4 discusses the experiments and results.  Section 5 consists of the discussion; finally, in Section 6, the research work is concluded.

## 2. Related Work

Currently, the diagnosis of molecular subtypes of breast tumor is mainly based on surgical or puncture biopsy immunohistochemistry, which is the gold standard for the detection of ER, PR, HER-2, and Ki-67 expression, and the reliability of its tests also depends on the handling of the tissue, which may sometimes lead to false positives and false negatives [15]. Therefore, predicting the molecular subtype of breast tumor by imaging signs can further improve the reliability of preoperative treatment strategies, which is of great value for the precise treatment of breast tumor and improving the prognosis. With the development of imaging technology in recent years, DBT technology has played an important role in the diagnosis of breast tumor. DBT can clearly show the morphology, margins, and relationship with surrounding tissues of the lesion [16]. A simple lump is the most common and direct manifestation of breast tumor, and the results of this paper show that the majority of breast tumors present as simple lumps, with the main molecular subtype being luminal A. Burrs are a characteristic feature of invasive breast tumor, and their formation may be related to tumor pulling on the normal Cooper ligament or tumor cells infiltrating the surrounding tissue [17]. [18] found that 71% of burr masses in 317 breast tumor patients in DM were luminal A. Luminal A was 10.3 times more likely to show burr-like masses on radiographs than other subtypes, so luminal A correlated with burr-like mass margins. [19] found that burrs on the margins of the mass were 3.77 times more likely to be luminal A than those without burrs, and that burrs did not correlate significantly with luminal B. This means that burrs are strongly associated with luminal A breast tumor. In this paper, the predominance of masses with burrs on the margins in luminal A is generally consistent with the results of the literature, and DBT is of great value in showing the boundaries of masses, especially malignant masses with burrs. DBT was shown to be able to see roughly 77 percent of the boundaries of a displayable mass in [20], whereas DM could only see about 53 percent of the boundaries.

The article "The Effect of PACS in Breast Tumor Diagnosis Based on Numerical Analysis" was published in 2022. Journal: Comput Math Methods Med.

In the study by [18], HER-2 types were most frequently seen as masses with calcification, followed by calcification alone, which is consistent with the results of this paper. [19] reported that breast tumors with HER-2 expression or amplification in molecular subtypes are more aggressive and difficult to treat, and malignant calcifications are more likely to develop in patients with HER-2 expression or amplification breast tumor. However, it has also been shown [20] that the presence of malignant calcification in breast tumor is not only associated with HER-2 expression or amplification but may also be related to other factors such as hormonal expression status. The results of this paper show that calcification is mainly seen in HER-2 expressing types and that DM combined with DBT does not improve the detection of calcification. However, it has also been reported that due to the abundance of glands in the breast, micro calcifications may be masked and DBT may reduce the interference of overlapping glands and improve the detection of calcifications.

In summary, the results of this paper suggest that DM combined with DBT is predictive of molecular subtypes of breast tumor and that certain imaging signs may be useful for preoperative individualization of treatment strategies and prognostic assessment.

## 3. Materials and Methods

### 3.1. General Information

Patients with breast tumor attending our hospital were selected. A total of 20 patients with 15 lesions were included in the analysis, all were female, aged 33-75 years, with a mean age of 52.6 ± 10.3 years. Inclusion criteria are as follows: (1) patients with breast tumor confirmed by puncture biopsy or surgical pathology and (2) mammography and DBT were performed before biopsy or surgery. Exclusion criteria are as follows: the quality of the images did not meet the diagnostic requirements. This work was approved by our hospital.

The article "The Effect of PACS in Breast Tumor Diagnosis Based on Numerical Analysis" was published in 2022. Journal: Comput Math Methods Med.

### 3.2. Inspection Methods

The Siemens Mammomat Inspiration completely digital mammography equipment is used to perform mammography in the craniocaudal (CC) and mediolateral oblique (MLO) orientations. In each case, a single DM position is obtained, followed by an automatic DBT scan under the same compression conditions, in which the X-ray bulb is rotated over the breast and the breast is scanned from -25° to 25°, with automatic exposure every 2° of rotation, to obtain multiple low-dose X-ray images at different angles. The glandular thickness of the compressed breast determines the number of layers.

### 3.3. Image Analysis

The films were independently reviewed by two breast diagnosticians with associate or higher titles, and a consensus was reached after consultation. Breast tumor is described and evaluated on digital X-rays using the American College of Radiology's Breast Imaging Reports and Data (BI-RADS) standard, which assesses the different imaging presentations of breast tumor, including masses, calcifications, masses with calcifications, and structural distortions.

## 4. Results

### 4.1. General Comparison

A total of 20 lesions were found in 15 breast tumor patients, of which 13 (35.5%) were luminal A. Radiographs showed 13 (54.3%) simple masses and 7 (23.7%) masses with calcification. The difference in the percentage of different molecular subtypes was statistically significant (*P* < 0.05), as shown in Table 1. Simple masses were the most common among the molecular subtypes, especially luminal A. The percentage of calcification alone was higher in the HER-2 overexpressing type, with 35 cases of calcification alone and 20 cases of HER-2 overexpressing type (57%), a statistically significant difference compared with the other three types (*P* < 0.05). The margins of the masses were classified as clear, blurred, microlobulated, and burr-like (Figures 1–3), and the difference in the percentage of different molecular subtypes was statistically significant (*P* < 0.05), as shown in Table 2. The difference in the percentage of masses with clear margins was higher in the triple-negative type; the difference in the percentage of masses with indistinct margins was not statistically significant among the subtypes. The difference between PACS combined with DBT was statistically significant (*P* < 0.05), especially for masses with burr-like margins, as shown in Table 3 and Figures 1–3 showing specific examples.

Figures 1(a) and 1(b) are mammograms showing disorganisation of the external superior structures of the right breast with localised nodular changes. Figures 1(c) and 1(d) are mammograms of the breast.

The tomosynthesis shows a well-defined mass with segmental distribution of polymorphic calcifications. Triple negative invasive ductal carcinoma.

The article "The Effect of PACS in Breast Tumor Diagnosis Based on Numerical Analysis" was published in 2022. Journal: Comput Math Methods Med.

Figures 3(a) and 3(b) are mammograms showing a right supratentorial nodule with poorly defined margins. Figures 3(c) and 3(d) are tomosynthesis images of the mammary gland showing small nodules with well-defined margins and burrs. The nodules have well-defined margins with burrs and clearer signs of malignancy.

### 4.2. Comparison of Clinical Features

Benign breast tumors: MRI pattern is round, oval, or lobulated; uniform density; smooth, sharp margins; surrounding tissue shows halo signs, compression pushing; CT shows irregular or oval shape; well-defined borders; lobulated masses with burrs; tumor is denser than the gland on plain scan, but more clearly outlined on enhanced scan. Breast tumor: MRI is lobulated, nodular, or irregular; uneven density, infiltrative margins, burrs, surrounding invasion, irregular edematous bands, irregular margins; CT shows a confined lamellar lesion in the breast with no obvious mass shadow, higher density than the surrounding gland, unclear borders, significant calcification; infiltrative patients show flattened dense areas throughout the gland, with pinpoint edges of varying length.

The detection rate of breast tumor by MRI and CT was 95.21% and 96.37%, sensitivity was 98.74% and 98.21%, and specificity was 52.34% and 54.23%, with no statistically significant difference (*P* > 0.05); see Tables 4 and 5.

There was no statistically significant difference between CT and MR in the detection rates of LDC and IDC (*P* > 0.05); see Table 6.

## 5. Discussion

PACS is an important adjunct to the early diagnosis of breast tumor in clinical practice, as it can provide multisequence, multiparameter, multidirectional imaging with high soft tissue resolution and can effectively differentiate between benign and malignant tumors. In this study, 90 of the 98 patients with PACS-diagnosed breast tumors were ultimately diagnosed as breast tumors after pathological histological investigation or surgery, while the remaining eight cases were benign tumors.

Most breast tumors appear as irregular low-signal masses at T1W1, while at T2W1, they appear as enhanced signals. The signal characteristics of the tumor are related to the internal composition of the tumor; the more collagen fibres the cells have, the more water they contain and the more pronounced their signal. Mucinous adenocarcinoma shows high signal due to the large amount of mucus and low signal due to calcification and collagen degeneration in the hard interstitium. Because the tumor tissue is not clearly distinguished from the lesion tissue due to congestion, oedema, and surrounding infiltration, oedematous bands with stellate borders might be seen. In cases of tumor invasion of the Cooper Tropic or skin, local indentation, or thickening of the skin, involvement of the nipple and milk ducts may be observed. The pectoralis major muscle and fascia may be involved when the tumor is more advanced. However, PACS has its limitations and is not good at detecting significant calcification in the lesion.

The article "The Effect of PACS in Breast Tumor Diagnosis Based on Numerical Analysis" was published in 2022. Journal: Comput Math Methods Med.

PACS has an important application in tumor diagnosis because of its high spatial and density resolution. In this study, the tumor density was slightly higher than that of the gland on PACS plain scan, and the PACS values were more variable on enhanced scan, which is consistent with previous studies, due to the abnormal metabolism of breast tumor, the varying degree of development, and the high iodine uptake by tumor cells [21].

The irregular shape of the tumor, with infiltrative growth and raised burr margins, often associated with lobular hyperplasia or dense mammary glands, makes it difficult to distinguish the mass from normal tissue and hyperplastic glands, which is also a major factor in misdiagnosis on CT. In this study, the diagnostic accuracy, sensitivity, and specificity of CT for breast tumor were 96.67%, 96.67%, and 54.54%, with five cases being misdiagnosed, and the misdiagnosis rate was slightly higher than that of PACS. In the remaining two cases, the extent of enhancement may be lower than the actual extent of cancer due to the strong dependence of cancer enhancement on tumor vascularity. In the present study, the detection rate of DCIS was statistically higher on CT than on MRI (*P* < 0.05), while the detection rates of LDC and IDC on PACS were not statistically different (*P* > 0.05).

DCIS is a malignant proliferation of epithelial cells in the ductal system of the breast, which is characterized microscopically by a poorly defined peribasal stromal infiltration.

## 6. Conclusions

However, PACS is not suitable for patients with metal prosthesis, pacemakers, obesity, and claustrophobia, while CT requires a certain amount of X-ray irradiation and may cause radiation damage. Furthermore, certain patients who are allergic to contrast chemicals are not candidates for PACS; thus, the clinical practice can select the most appropriate examination approach based on the patient's current circumstances in order to increase the lesion's detection rate. The accuracy and sensitivity of the test can also be improved by combining the tests.

## Figures and Tables

**Figure 1:** Female, 63 years old. Luminal type B invasive ductal carcinoma.

**Figure 2:** (a) and (b) are mammograms. The mammogram shows an upper middle breast mass with poorly defined margins. (c) and (d) are tomosynthesis images of the breast showing radiolucent burrs around the mass with clear signs of malignancy.

The article "The Effect of PACS in Breast Tumor Diagnosis Based on Numerical Analysis" was published in 2022. Journal: Comput Math Methods Med.

**Figure 3:** Female, 68 years old. Luminal type A invasive ductal carcinoma.

**Table 1:** Comparison of different molecular subtypes of X-ray lesion types.

Mass margin	Luminal type A	Luminal type B	HER-2 overexpression	Three yin types	*x* ^2^	*P*
Simple mass	5	7	9	4	1.247	<0.001
Mass with calcification	6	3	4	3		
Simple calcification	7	2	1	0		
Structural distortion	1	9	2	0		

**Table 2:** Comparison of the margins of the masses on X-rays with different molecular typing.

Mass margin	Luminal type A	Luminal type B	HER-2 overexpression	Three yin types	*x* ^2^	*P*
Clear edge	6	7	0	2	5.257	<0.001
Edge blur	1	2	4	9		
Differential leaf	3	1	5	2		
Skin needling	3	2	3	2		

**Table 3:** Comparison of DM and DM combined with DBT image features.

		DM	DM+DBT	*x* ^2^	*P*
Lesion type	Simple mass	6	3	1.124	<0.001
	Mass with calcification	2	5	2.024	0.002
	Simple calcification	1	3	0.270	0.541
Mass margin	Clear edge	2	2	2.234	0.039
	Edge blur	2	5	5.471	<0.001
	Differential leaf	1	3	3.958	0.001
	Prickly	4	1	1.587	0.001

**Table 4:** Comparison of MRI and CT diagnostic findings with pathological procedures (cases).

Surgical pathology	MRI		Total
	Positive	Negative	
Positive	4	6	10
Negative	1	7	8
98 total	5	3	8

Surgical pathology	CT		Total
	Positive	Negative	
Positive	5	5	11
Negative	2	6	8
98 total	7	1	8

**Table 5:** Value of MRI and CT in breast tumor (%).

Inspection method	Detection rate	Sensitivity	Specificity
MRI	95.210	98.740	52.340
CT	96.370	98.210	54.240
*x* ^2^ value	0.101	10123	0.114
*P* value	0.785	0.814	0.797

**Table 6:** MRI and CT in different types of breast tumor (%).

Inspection method	Detection rate	Pathological type		
		DCLS	LDC	IDC
MRI	92.24	85.74	100	100
CT	95.37	100	95.710	96.210

## Data Availability

The dataset used in this paper are available from the corresponding author upon request.
